# Clinical Efficacy of Chinese and Western Medicine in the Treatment of Benign Thyroid Nodules: A Meta-Analysis

**DOI:** 10.1155/2022/3108485

**Published:** 2022-05-28

**Authors:** Yu Zhu, Ju Huang, Rensong Yue, Tao Shen

**Affiliations:** Hospital of Chengdu University of Traditional Chinese Medicine, Chengdu 610072, China

## Abstract

**Background:**

Studies have shown that Chinese herbal medicine (CHM) effectively improved the response rate and reduced the maximum nodule diameter of benign thyroid nodules (BTN). This study aimed at systematically reviewing all related studies to assess the clinical efficacy of CHM and Western medicine in the treatment of BTN.

**Methods:**

PubMed, Web of Science, Embase, China National Knowledge Infrastructure, and Wanfang databases were searched for randomized controlled trials, published between 2000 and 2021, on CHM for treating BTN. The control group comprised patients treated with Western medicine (oral thyroxine tablets or microwave ablation), while the treatment group was treated with CHM combined with Western medicine. Meta-analysis was performed using the Stata 16.0 software.

**Results:**

A total of 264 articles were retrieved, of which 12 were finally selected for analysis after screening. The results showed that combined therapy was associated with a higher response rate (OR = 3.35, 95% CI (2.40, 4.68), *P* < 0.05). After treatment, the maximum nodule diameter (SMD = −0.76, 95%, CI (−0.98, −0.53), *P* < 0.05) and thyroid volume (SMD = −1.14, 95%, CI (−1.94, −0.35), *P* < 0.05) of the treatment group were smaller than those of the control group. Furthermore, the combined treatment was associated with lower levels of free triiodothyronine (FT3), free thyroxine (FT4), and thyroid-stimulating hormone (TSH) in the serum of patients and lower traditional Chinese medicine (TCM) syndrome score (SMD = −1.87, 95%, CI (−3.16, −0.58), *P* < 0.05).

**Conclusion:**

CHM combined with thyroid hormone/microwave improved the response rate of BTN. The combined treatment was also associated with reducing the maximum nodule diameter, thyroid volume, levels of FT3, FT4, and TSH, and TCM syndrome score. Therefore, combining CHM with WM could be considered as an alternative and effective treatment for treating BTN, suggesting promising integration of Chinese medicine with Western medicine.

## 1. Introduction

Thyroid nodule (TN), caused mainly by abnormal local growth of thyroid cells, is a common disease in surgery [1]. Clinically, thyroid degeneration, autoimmunity and inflammatory reaction, and other thyroid diseases can be characterized as nodules and mainly present as a nodular goiter or inflammatory nodules [2]. Based on its degree of differentiation, TN can be divided into benign and malignant nodules, with the former representing the majority of TN cases [3]. In recent years, the detection rate of TN has been increasing on a yearly basis, which could be related to changes in the living environment, economic growth, elevated health awareness, and advances in medical technology [4]. For the general population, the detection rate of TN by palpation ranges from 3% to 7%, whereas that by high-frequency ultrasound ranges from 20% to 76%.

Currently, only about 5% to 15% of TNs are malignant [5, 6]. Considering that the American Thyroid Association Management guidelines suggest that the probability of benign thyroid nodules (BTNs) undergoing malignant transformation is extremely low [7], it would be too invasive to perform surgeries to treat BTN. However, apart from surgery, there is no widely used effective therapy for BTN [8].

In China and many other countries, Chinese herbal medicines (CHMs) have been used by traditional Chinese medicine (TCM) practitioners to treat many diseases [2–4]. In TCM, TN can be prevented and treated using various methods and could be associated with advantages such as fewer adverse reactions [5, 6]. TCM considers the occurrence of TN to be related to changes in the environment, diet, and personal emotions. Considering that TCM is a form of personalized treatment, treatments for BTN are usually based on its etiology, pathogenesis, syndrome characteristics, and patients' conditions [4]. Thus, the type of CHM used can vary depending on the TCM syndromes of the patients. In CHM, TN has been treated using Sanjie Pingying, Codonopsis Pilosula, Figwort root, Pangolin Scales, Self-Heal, Chinese Thorowax root, Nutgrass Galingale Rhizome, Seaweed, Laminaria Tents, and others [3, 4, 9–11]. According to theories of TCM, TCM practitioners recognize that TN is caused by blood stasis, Qi stagnation, and phlegm coagulation. Thus, most of the prescriptions used to treat BTN are often a combination of self-made prescriptions, and the drugs that are used mainly target issues such as resolving phlegm, soothing the liver, regulating qi, and clearing of blood stasis.

Studies based on TCM have shown that CHM could shrink TN without significant adverse events [3, 9, 10]. Furthermore, in recent years, a number of clinical studies have confirmed that Chinese herbal medicine (CHM) decoction alone or in combination with Western medicine (WM) could effectively treat BTN by reducing their maximum diameter [9–11]. However, current studies have mostly been single-centered studies with small sample sizes, limiting the evidence level of their findings. A systematic evaluation of external therapy of CHM in the treatment of BTN is still lacking.

In this study, we aimed at performing a meta-analysis to analyze the outcomes of CHM and Western medicine in treating BTN using data from existing randomized controlled trials (RCTs) to provide a higher level of evidence for the clinical treatment of BTN.

## 2. Materials and Methods

### 2.1. Strategies for Literature Retrieval

Relevant studies published between 2000 and 2021 were retrieved from PubMed, Web of Science, Embase, China National Knowledge Infrastructure, and Wanfang database. The English and Chinese search terms used included (#“1Traditional Chinese medicine/Chinese medicine”) and (#“2Treatment”) and (3“Benign thyroid nodule,”) and (#4“Clinical efficacy”).

### 2.2. Selection Criteria

Studies were selected for final analysis based on the following criteria: (1) study subjects: patients diagnosed with BTN by traditional Chinese medicine (TCM) and WM; (2) intervention measures: patients in the control group were treated with oral thyroxine tablets or microwave ablation, while those in the treatment group were treated with at least one Chinese herbal formula in combination with WM; (3) outcome measures (with at least one of the following indicators): these contained sufficient data to assess the treatment response rate, maximum nodule diameter, thyroid volume (TV), posttreatment free triiodothyronine (FT3) levels, posttreatment free thyroxine (FT4) levels, posttreatment thyroid-stimulating hormone (TSH), and the TCM syndrome score [12]; (4) study type: RCTs.

Studies were excluded based on the following criteria: (1) studies contained duplicated or lacked sufficient data for assessing the outcomes of measures required for this meta-analysis; (2) full text could not be retrieved; (3) studies were reviews, case reports, letters, conference papers, or contained animal experiments.

### 2.3. Data Extraction

Literature screening was independently performed by two reviewers, who extracted and recorded the data following the study's inclusion and exclusion criteria. Data extracted included the following: (1) name of authors from the retrieved studies; (2) year of publication; (3) sample size in the control and treatment groups; and (4) outcome measures. Disagreements were resolved by a mutual consensus between the two reviewers or by consultation with a third reviewer. If necessary, the authors of the included articles were contacted to obtain important data that were not mentioned in the retrieved literature.

### 2.4. Statistical Analysis

Data were analyzed using the Stata 16.0 software. First, the *χ*^2^ test was conducted to test the heterogeneity of the selected studies, using a test level *α* = 0.05. If no significant heterogeneity was found (*I*^2^ < 50% and *P* > 0.10), the fixed-effects model was used to combine the effect sizes; otherwise, the random-effects model was used. Furthermore, the stability of the overall results was tested by sensitivity analysis. Funnel plots and Begg's test were adopted to evaluate publication bias. The standard mean difference (SMD) was used as a measure for data measurement, while the odds ratio (OR) and 95% confidence interval (CI) were used for categorical variables. For *P* < 0.05, the difference between comparisons was considered statistically significant.

## 3. Results

### 3.1. Results of Literature Retrieval

In total, 264 studies were retrieved following the search strategies. At initial screening, 203 articles were excluded based on the study criteria. Then, after examining the full text of the remaining studies, only 12 RCTs were found eligible for this meta-analysis [9–20]. The literature screening process is illustrated in Figure 1. The characteristics of the included studies are shown in Table 1.

### 3.2. Meta-Analysis of the Treatment Response Rate

Eleven studies [9–11, 13–20] had response rate data for the two treatment groups. No significant heterogeneity (*I*^2^ = 0.0%, *P*=0.867) was found among the studies, so the fixed-effects model was employed to combine the effect size. Our results showed that the response rate of the treatment group was significantly higher than that of the control group (OR = 3.35, 95% CI (2.40, 4.68), *P* < 0.05; Figure 2(a)).

The funnel plot showed some level of asymmetries, suggesting potential publication bias in the included studies, which could have been due to negative results of the included studies (Figure 2(b)). Sensitivity analysis was performed, and the corresponding literature was removed one by one. The findings showed that the article by Wang and Li [10] might be the primary source of heterogeneity. The results obtained after the exclusion of this article were still consistent with those before exclusion (Figure 2(c)). Hence, the overall results of this present study can be considered relatively stable and reliable.

### 3.3. Meta-Analysis of the Maximum Thyroid Nodule Diameter and Thyroid Volume after Treatment

The effects of combined CHM and Western medicine on the maximum nodule diameter have been stated in seven studies [9–14, 16], while five studies [10, 13, 14, 18, 20] had data for assessing the TV. Heterogeneity was found among the included studies regarding the two indicators, respectively (all *I*^2^ > 50%, *P* < 0.05), so the random-effects model was used to combine the effect size. The results showed that the maximum nodule diameter (SMD = −0.76, 95%, CI (−0.98, −0.53), *P* < 0.05; Figure 3(a)) and TV in the treatment group were significantly smaller than those in the control group (SMD = −1.14, 95%, CI (−1.94, −0.35), *P* < 0.05; Figure 3(b)).

Sensitivity analyses were performed due to heterogeneity observed among the included studies. Based on the obtained results, by eliminating one by one, we observed that the studies by Wang and Li [10] and Mou [12] might have been the main source of increased heterogeneity. By excluding these two studies, the results still suggested that the treatment group had a smaller maximum nodule diameter after treatment (Figure 4(a)). Again, after excluding the studies from Liu et al. [18] and Qiu [20], the obtained results still showed that the TV of the treatment group was smaller than that of the control group after treatment (Figure 4(b)). These findings suggest that the overall analysis of this study was relatively stable and reliable.

### 3.4. Meta-Analysis of Hormone Levels after Treatment

Five studies [11–14, 19] reported the effects of combined CHM and Western medicine on FT3, FT4, and TSH levels. As heterogeneity was observed among the included studies in terms of FT3 (*I*^2^ = 55.1%, *P*=0.063), FT4 (*I*^2^ = 93.3%, *P* < 0.001), and TSH (*I*^2^ = 95.9%, *P* < 0.001) (Figures 5(a)–5(c)), the random-effects model was used to combine the effect sizes. Our findings showed that the treatment group had lower levels of these three indicators. Specifically, compared with the control group, the levels of FT4 (SMD = −0.33, 95%, CI (−0.39, 1.05), *P* < 0.05) and TSH (SMD = −1.34, 95%, CI (−2.34, −0.35), *P* < 0.05) were significantly lower in the treatment group, while no significant difference between the two treatment groups was observed for FT3 levels (SMD = −0.22, 95%, CI (−0.39, −0.04), *P*=0.063).

Sensitivity analyses were performed, and the results showed that the study by Mou [12] might be primarily responsible for the heterogeneity observed when analyzing FT3, FT4, and TSH levels. After excluding this study, the findings showed that the levels of FT3, FT4, and TSH in the treatment group were lower than those in the control group (Figures 6(a)–6(c)).

### 3.5. Meta-Analysis of the Traditional Chinese Medicine Syndrome Score after Treatment

The TCM syndrome score was calculated based on the retrieved data. A higher score refers to a more severe disease [12]. Of the retrieved literature, 4 studies [12, 13, 16, 19] compared TCM syndrome scores after treatment between the two treatment groups. The random-effects model was used to combine the effect size (*I*^2^ = 96.8%, *P* < 0.001) (Figure 7(a)), and the corresponding findings indicated that the TCM syndrome score of the treatment group was significantly lower than that of the control group (SMD = −1.87, 95%, CI (−3.16, −0.58), *P* < 0.05). Sensitivity analysis was performed, and the results showed that the study of Wang et al. [19] might have been the primary cause for the heterogeneity observed between the studies when analyzing TCM syndrome scores. After excluding this paper, the results obtained showed that the TCM syndrome score of the treatment group was still lower than that of the control group (Figure 7(b)).

## 4. Discussion

TN is a common disease for which treatment is mainly based on surgery, internal medicine, and nuclear medicine. Of all TNs diagnosed, only 5–15% are malignant and are primarily found in females [21]. In recent years, thyroid cancer has emerged as one of the most commonly seen malignant tumors as the incidence of TN has been increasing year by year [22]. At present, treatment of TN includes regular follow-up, conventional surgery, TSH suppressive therapy, radioiodine therapy, percutaneous ethanol injection therapy, laser ablation, radiofrequency ablation, and microwave ablation [23].

Considering that the number of BTN patients has been increasing clinically and the limitations often observed in the existing treatment methods, more and more scholars in China and abroad have investigated the effects of CHM therapy on BTN. Based on favorable clinical results, CHM therapy for TN has acquired widespread recognition in the academic community. Yu and Xu [24] found that Xiaoliu Decoction No. 1, made by Professor Xu Bin, could effectively treat TN by reducing its maximum nodule diameter and TCM syndrome score. Based on a study by Lin [25], the Haizao Yuhu Decoction was found to effectively decrease the diameter and cross-sectional area of TN. In a study by Huang and Ma [26], the authors found that BTN could be effectively treated through TCM by regulating qi, resolving phlegm, and targeting blood stasis. In regard to reducing TV and improving the symptoms and signs of patients with BTN, these studies suggested that CHM could have better treatment outcomes than traditional therapy in treating BTN. Hence, we performed this systematic analysis to assess the clinical efficacy of CHM in treating BTN. Overall, the results of this meta-analysis showed that, compared with WM alone, CHM decoction combined with WM had better treatment response rates. Besides, the combined therapy could effectively reduce the maximum diameter of BTN and achieve significant decreases in FT3, FT4, and TSH levels and TCM syndrome scores. These findings provide credible evidence for the clinical application of CHM therapy in treating BTN.

Although promising results in using CHM to treat BTN were observed, there were still some important limitations. All the literature selected for this study was retrieved using electronic database searches and manual screenings, which could have led to unintentional omission of some potentially eligible studies due to deficiencies in the strategies or the database used; (2) heterogeneities observed in this study could not be avoided due to differences in drugs, dosage, administration frequency, and treatment course in the included RCTs retrieved; (3) the included studies were from only one country (China), and the quality of these RCTs was not very high, which might have caused certain levels of bias in the statistical results. Therefore, cross-population multicenter RCTs with larger samples are still required to further confirm the role of CHM in treating TN.

## 5. Conclusion

In summary, CHM combined with thyroid hormone or microwave ablation was superior to WM alone in improving the clinical symptoms of BTN patients. The combined therapy was also found to effectively soften and dissipate nodules and promote the recovery of thyroid function. Thus, these results support that the integration of Chinese medicine with WM could be a clinically viable treatment alternative for treating BTN.

## Figures and Tables

**Figure 1:** Flow chart of literature screening.

**Figure 2:** Meta-analysis of the efficiency of combined Chinese and Western medical treatment modalities in patients with thyroid nodules. (a) Forest plot of treatment response rate. (b) Funnel plot of treatment response rate. (c) Sensitivity analysis of treatment response rate.

**Figure 3:** Meta-analysis of the maximum nodule diameter and thyroid volume in patients with thyroid nodules treated with a combination of Chinese and Western medicine. (a) Forest plot of the maximum nodule diameter. (b) Forest plot of thyroid volume.

**Figure 4:** Sensitivity analysis of the maximum nodule diameter and thyroid volume in patients with thyroid nodules treated with a combination of Chinese and Western medicine. Sensitivity analysis of the maximum nodule diameter (a) and thyroid volume (b).

**Figure 5:** Meta-analysis of hormone levels in patients with thyroid nodules treated with a combination of Chinese and Western medicine. Forest plot of serum FT3 (a), FT4 (b), and TSH levels (c) after treatment.

**Figure 6:** Sensitivity analysis of hormone levels in patients with thyroid nodules treated with a combination of Chinese and Western medicine. (a) Sensitivity analysis of serum FT3 levels after treatment. (b) Sensitivity analysis of FT4 levels after treatment. (c) Sensitivity analysis of TSH levels after treatment.

**Figure 7:** Meta-analysis of the TCM syndrome score in patients with thyroid nodules treated with a combination of Chinese and Western medicine. (a) Forest plot of the TCM syndrome score of patients after treatment. (b) Sensitivity analysis of the TCM syndrome score of patients after treatment.

**Table 1:** Basic characteristics of the literature reporting on benign thyroid nodules included for this meta-analysis.

Study	Year	Sample time (year.month)	Cases treat/con	Age (years)		Sex (male/female)		Follow-up time	Study design	Outcome measures
				Treat group	Con group	Treat group	Con group			
Jiang Hongyu	2004	2002.05–2003.05	43/30	39.9 ± 14.3	40.4 ± 16.3	16/27	7/23	3	RCT	(1)(2)
Fu Lijuan	2020	2018.10–2019.10	78/78	65.4 ± 21.6	10.7 ± 7.3	38/40	39/39	6	RCT	(1)
Liu Yong	2021	2019.01–2019.12	42/42	65.4 ± 21.6	65.4 ± 21.7	23/19	24/18	6	RCT	(1)(3)
Wang Leilei	2014	2010.07–2012.12	95/90	51.4 ± 8.2	50.9 ± 8.5	21/74	19/71	6	RCT	(1)(2)(3)
Wang Junlin	2021	2018.10–2019.10	78/78	31–86	31–86	38/40	39/39	6	RCT	(1)(4)(5)(6)(7)
Lin Min	2020	2019.01–2019.06	30/30	NR	NR	NR	NR	3	RCT	(1)(2)(4)(5)(6)
Mou Linan	2017	2014.10–2015.10	30/30	43.1 ± 4.9	42.9 ± 4.1	10/20	11/19	2	RCT	(2)(4)(5)(6)(7)
Tong Rui	2020	2018.02–2019.02	52/52	41.5 ± 7.4	43.8 ± 7.2	11/41	13/39	6	RCT	(1)(2)(3)(4)(5)(6)(7)
Shen Yuguo	2018	2014.06–2016.06	62/63	29–54	29–54	20/42	20/43	6	RCT	(1)(2)(3)(4)(5)(6)
Liu Wenxiu	2019	2015.02–2018.02	74/71	47.1 ± 10.7	46.5 ± 11.4	24/50	22/49	6	RCT	(1)
Qiu Jintao	2020	2017.06–2019.10	30/30	41.3 ± 10.8	42.4 ± 9.7	6/24	4/26	6	RCT	(1)(3)
Zhang Lili	2018	2017.01–2017.09	68/68	42.2 ± 5.9	42.6 ± 5.4	23/45	24/44	6	RCT	(1)(2)(7)

*Note.* Treat: treatment; con: control; RCT: randomized controlled trial; NR: not reported; (1) effective rate; (2) maximum nodule diameter; (3) thyroid volume (TV); (4) free triiodothyronine (FT3); (5) free thyroxine (FT4); (6) thyroid-stimulating hormone (TSH); (7) traditional Chinese medicine syndrome score.

## Data Availability

The data used to support the findings of this study are available from the corresponding author upon request.
